# Dynamic Total-Body PET/CT Imaging Reveals Kinetic Distribution of ^68^Ga-DOTATATE in Normal Organs

**DOI:** 10.1155/2023/4722499

**Published:** 2023-01-18

**Authors:** Hongyan Yin, Guobing Liu, Yan Hu, Jie Xiao, Wujian Mao, Jing Lv, Haojun Yu, Qingyu Lin, Dengfeng Cheng, Hongcheng Shi

**Affiliations:** ^1^Department of Nuclear Medicine, Zhongshan Hospital, Fudan University, Shanghai 200032, China; ^2^Institute of Nuclear Medicine, Fudan University, Shanghai 200032, China; ^3^Shanghai Institute of Medical Imaging, Shanghai 200032, China; ^4^Cancer Prevention and Treatment Center, Zhongshan Hospital, Fudan University, Shanghai 200032, China

## Abstract

**Objective:**

To investigate the biodistribution and kinetic constants of ^68^Ga-DOTATATE in normal organs through dynamic total-body positron emission tomography/computed tomography (PET/CT).

**Methods:**

Seven patients who experienced endoscopic resection of gastric neuroendocrine tumor were enrolled. Dynamic total-body PET/CT scans over 60 min were performed. Time-activity curves were obtained by drawing regions of interest in normal organs. Rate constants, including *K*_1_, *k*_2_, *k*_3_, and vB, were computed using a two-tissue compartment model. Factor analysis was used to compare the rate constants among subjects and regions. Hierarchical cluster analysis was performed to identify organs with similar kinetic characteristics.

**Results:**

The highest uptake of ^68^Ga-DOTATATE was observed in the spleen followed by kidneys, adrenals, liver, pituitary gland, pancreas head, prostate, pancreas body, and thyroid, parotid, and submandibular glands. Low background level of ^68^Ga-DOTATATE uptake was observed in the nasal mucosa, bone, blood pool, and cerebrum. In addition, the uptake in the pancreas head was noted to be higher than the pancreas body (*P* < 0.001) on the basis of each time point of dynamic PET. There were differences of rate constants among different organs. The mean *K*_1_ ranged from 0.0507 min^−1^ in the left nasal mucosa to 1.21 min^−1^ in the left kidney, and mean *k*_2_ ranged from 0.0174 min^−1^ in the spleen to 4.4487 min^−1^ in the left cerebrum. The mean *k*_3_ ranged from 0.0563 min^−1^ in the right cerebrum to 4.6309 min^−1^ in the left adrenal, and mean vB ranged from 0.0001 in the left cerebrum to 0.2489 in the right adrenal. However, none of the rate constants was significantly different among subjects or among different sites within a single organ. Three groups of organs with similar kinetic characteristics were identified: (1) cerebrum; (2) pituitary gland, liver, adrenal, and prostate; and (3) nasal mucosa, parotid and submandibular glands, thyroid, spleen, pancreas, kidney, and bone.

**Conclusion:**

Uptake and clearance of ^68^Ga-DOTATATE, in terms of kinetic constants, were different in different organs. The kinetic parameters of ^68^Ga-DOTATATE in different organs provide a reference for future dynamic PET imaging.

## 1. Introduction

Neuroendocrine tumors (NET) are heterogeneous neoplasms arising from neuroendocrine cells in different organs [1]. High somatostatin receptor (SSTR) expression of NETs allows ^68^Ga-somatostatin analog (SSA) positron emission tomography/computed tomography (PET/CT) imaging for diagnosis and treatment. Standardized uptake value (SUV) using in the traditional static PET image is a widely used semiquantitative marker of SSTR expression. However, changes of tumor SUV in ^68^Ga-DOTATOC PET imaging have been found no correlation with the treatment outcome in peptide receptor radionuclide therapy [2, 3].

By contrast, net uptake rate (*K*_*i*_) determined by tracer kinetic analysis of dynamic PET image appeared to be a more accurate measurement tool for quantification of SSTR density and therapeutic evaluation than those of SUV [4]. However, ^68^Ga-SSA dynamic PET/CT imaging studies have been limited mostly to tumors, such as meningiomas [5] and metastatic neuroendocrine tumors [4, 6–8]. As yet, few systematic studies about kinetic parameters of normal organs have been reported. This is mainly because previous dynamic protocols capture data within a very limited scan range, equivalent to the axial field-of-view of the traditional PET scanner (typically 15–30 cm). The recent introduction of a 194 cm long total-body PET/CT scanner allows simultaneous total-body dynamic imaging and high-quality tracer input function from major arteries, avoiding invasive arterial blood sampling [9].

A study of 2-deoxy-2-[^18^F]fluoro-D-glucose ([^18^F]FDG) kinetics in normal organs using total-body PET served as a reference for pharmacokinetic studies in other radiotracers [9]. Considering the ultra-high sensitivity of about 174 kcps/MBq [10], the author further demonstrated that dynamic [^18^F]FDG total-body PET scan with ultra-low activity obtained relevant kinetic metrics of full activity with the advantage of decrease in radiation dose and data size [11]. Although the administered dose of ^68^Ga-SSA is 2 MBq/kg of body weight [12], 1 MBq/kg of body weight was used in this study based on our previous total-body dynamic PET data. The aim of this study was to investigate the biodistribution and kinetic parameters of ^68^Ga-DOTATATE in normal organs through dynamic total-body PET/CT imaging with half-dose activity.

## 2. Materials and Methods

### 2.1. Patients

This prospective study was approved by the Institutional Review Board of Zhongshan Hospital, Fudan University (approval number IRB-B2020-186R), and all patients signed informed consent. The patients had only undergone endoscopic resection for gastric neuroendocrine tumor (gNET) earlier without other therapy and had been referred for ^68^Ga-DOTATATE PET/CT to search for evidence of residual or metastatic disease from August to December 2020. Seven patients were included in this study based on the following criteria: (1) no evidence of recurrent disease on conventional imaging before ^68^Ga-DOTATATE PET/CT, (2) all patients underwent 60 min dynamic PET imaging, and (3) no tracer-avid recurrence and metastases on PET scan. Detailed information of the seven patients is shown in Table 1.

### 2.2. Total-Body Dynamic PET/CT Imaging

^68^Ga-DOTATATE was prepared as described previously [13]. Total-body PET/CT (uEXPLORER, United Imaging Healthcare, Shanghai, China) with an axial field-of-view of 194 cm was used in this study. The patient first underwent a low-dose CT scan (120 kV; 10 mAs) over total body for attenuation correction. Then, 60 min dynamic PET scanning was performed simultaneously after a bolus injection of 48.1–73.6 MBq ^68^Ga-DOTATATE by hand into a vein near the ankle. At the end of the dynamic acquisition, a high-dose CT scan from head to proximal femoral was performed (120 kV; automatic tube current modulation) for diagnosis. The PET images were corrected for attenuation, scatter, alignment, decay, normalization, and randoms. Then, they were reconstructed using list-mode ordered subset expectation maximization (three iterations, 20 subsets) algorithm incorporating time-of-flight and point spread function modeling applying a 3.0 mm Gaussian filter. The image matrix size was 192 × 192 pixels. The dataset was divided into 55 frames: 36 × 5 s, 19 × 180 s. Representative frames of PET images are shown in Figure 1.

### 2.3. Time–Activity Curves (TACs)

Reconstructed PET and CT images were transferred to the vendor-provided workstation (uWS-MI R001; United Imaging Healthcare, Shanghai, China) for dynamic analysis. Two-dimensional regions of interest (ROIs) were drawn in organs according to the method described previously [9, 11]. ROIs were drawn at the same locations on the total-body images and on the last time frame of the dynamic scans, which were transferred to all earlier time frames. ROIs as large as possible were drawn within the limits of the activity distribution on PET, avoiding any obvious anatomical abnormalities or blood vessels on CT. ROI placement in each organ is shown in Figure 2.

The input function was obtained by drawing ROI in the ascending aorta as described by Liu et al. [9] because the ascending aorta is the closest major artery to the heart, and it is not affected by breathing and cardiac movements and the spillover of activity. Cerebrum ROIs were drawn in the temporal lobe on both sides to represent brain tissue as described previously [5]. For pituitary gland, ROI was placed in the middle of the gland. For the nasal mucosa, parotid and submandibular glands, thyroid, adrenal, and kidney cortex, ROIs were placed in the middle of each side. Liver ROIs were drawn in the upper, middle, and lower areas of the right lobe and middle area of the left lobe. Pancreas ROIs were drawn in the head and body part. Spleen ROI was placed in the area with the largest transaxial size. Prostate ROI was drawn in the middle of the gland. Bone ROI was placed in the third lumbar body. The average radioactivity concentration for each ROI was obtained at Bq/mL from each PET frames and TACs were generated for all organs.

### 2.4. Data Analysis

TAC data were uploaded to the PMOD software (version 3.201, PMOD Technologies Ltd., Zurich, Switzerland) [5–7]. The TAC data from the ROI in the descending aorta were used for image-derived input function (IDIF). A two-tissue compartment model was used for model fitting according to previous studies regarding dynamic ^68^Ga-DOTATOC PET imaging [5–7]. The default setting of PMOD regarding the lower and upper bounds of estimated kinetic parameter was applied, namely, 0–1 for vB and 0–8 for *K*_1_, *k*_2_, and *k*_3_. A constant weighting method with a factor of 0.05 was used. The rate constants *K*_1_, *k*_2_, and *k*_3_ and vB were computed. The compartmental configuration of this model is given in Figure 3. *K*_1_ is associated with the receptor binding, *k*_2_ with the displacement from the receptor, *k*_3_ with the cellular internalization, and *k*_4_ with the externalization. As *k*_4_ is commonly close to zero, it was not analyzed in this study [5, 14].

### 2.5. Statistical Analysis

Statistical analyses were conducted using SPSS software version 23.0 (IBM Corp., New York, NY, USA). If necessary, the summary statistic is expressed as mean ± standard deviation and coefficient of variation. Factor analysis was used to compare the rate constants of organs among subjects and regions. Variances were compared using mixed models. Hierarchical cluster analysis was performed to identify organs with similar kinetic characteristics. Significance was set at *P* < 0.05 and all *P*-values reported were two-sided.

## 3. Results

### 3.1. Patient Characteristics

Seven patients (five males, two females; age 39–68 years) were imaged. All tumors were low- to intermediate-grade gNET, according to the World Health Organization 2019 grading of gastroenteropancreatic NETs. Table 1 summarizes the patient characteristics. The mean injected activity of ^68^Ga-DOTATATE for all subjects was 65.6 ± 8.8 MBq.

### 3.2. Biodistribution

Figures 1 and 4 illustrate the biodistribution of ^68^Ga-DOTATATE as a function of time in normal organs. In the first few seconds after injection into a leg vein, the tracer traveled to the heart and was then distributed through the arteries to all the organs of the body. Gradual accumulation of the tracer could be seen in the kidneys, spleen, adrenals, liver, and pituitary, thyroid, and salivary glands. Clearance of ^68^Ga-DOTATATE from the blood was fast. Radioactivity in the blood decreased rapidly to 2.1% of the peak level within 60 min of the dynamic scanning after reaching the peak at 40 s. The highest uptake was observed in the spleen, adrenals, and pituitary gland, due to SSTR-specific uptake. High ^68^Ga-DOTATATE uptake in the kidneys and liver was also observed. Radioactivity in the spleen, adrenals, pituitary gland, and liver increased with time and no excretion trend was seen until 60 min. The rapid presence in the kidneys, followed by a passage toward the urinary bladder, illustrates the mainly renal excretion of the tracer. Limited uptake was also observed in the prostate and in the thyroid. Low background uptake was observed in the cerebrum and bone.

In addition, the uptake in the pancreas head was noted to be higher than the rest of the gland in the static PET image. Radioactivity of the pancreas head was significantly higher than that of the pancreas body (*P* < 0.001) on the basis of each time point of dynamic PET.

### 3.3. Kinetic Constants

The descriptive statistics of *K*_1_, *k*_2_, *k*_3_, and vB are shown in Tables 2 and 3. Representative fitted curves are shown in Figure 4. The rate constants varied widely between different organs. Mean *K*_1_ ranged from 0.0507 min^−1^ in the left nasal mucosa to 1.21 min^−1^ in the left kidney, and mean *k*_2_ ranged from 0.0174 min^−1^ in the spleen to 4.4487 min^−1^ in the left cerebrum. Mean *k*_3_ ranged from 0.0563 min^−1^ in the right cerebrum to 4.6309 min^−1^ in the left adrenal, and mean vB ranged from 0.0001 in the left cerebrum to 0.2489 in the right adrenal. There was no significant difference in the rate constants between different sites within an organ. The intersubject variances of *K*_1_ in various organs are acceptable. However, from *k*_2_ to *k*_3_, the intersubject variances showed an increasing trend. The largest intersubject variances in terms of CV for *k*_2_ and *k*_3_ were 264.6% in the left adrenal and 229.8% in the right middle area of liver, respectively. Furthermore, compared with the intersite variances of rate constants, the intersubject variances were larger and their contributions to the overall variances were remarkable, but was not statistically significant in any organ (*P* > 0.05). Mean *K*_1_, *k*_2_, and *k*_3_ values of the nasal mucosa were 0.0572, 0.1025, and 0.0771 min^−1^, respectively.

Figure 5 shows the distribution of organs in three-dimensional rate constant space and illustrates the maximum likelihood grouping. An optimum of three groups of organs was obtained, as shown in Table 4. The first group had the lowest *K*_1_ and *k*_3_, and the highest *k*_2_, representing low binding and internalization but high displacement of ^68^Ga-DOTATATE, and it consisted of the cerebrum. The second group consisted of the pituitary gland, liver, adrenal, and prostate, which had similar *K*_1_ values to those of organs from group 1, but with the lowest *k*_2_ and the highest *k*_3_, indicating low displacement and high internalization of ^68^Ga-DOTATATE. The third group had the highest *K*_1_ but a relatively lower *k*_2_ and *k*_3_, including the nasal mucosa, parotid and submandibular glands, thyroid, spleen, pancreas, kidney, and bone, indicating high binding but low internalization of ^68^Ga-DOTATATE.

## 4. Discussion

There are some important findings in this study. First, the biodistribution of ^68^Ga-DOTATATE in normal organs using dynamic total-body PET/CT imaging showed that the uptake and clearance in different normal organ types were different. Second, different kinetic characteristics were found in normal organs, which may reflect variable expression levels of SSTR. Besides, similar kinetic metrics were also found in some organs. The exact rationale for these findings is hard to explain, but there may be a reflection of the interorgan relationships in the kinetic metrics of ^68^Ga-DOTATATE in normal organs. As ^68^Ga-DOTATATE was considered stable without obvious metabolites in short time [4, 8], the kinetic metrics as identified in this study could be obtained with an IDIF noninvasively.

The 194 cm axial field-of-view of total-body PET/CT scanner has unique advantage over dynamic imaging. First, the scanner covers all organs in the body, and permits total-body dynamic imaging and kinetic analyses of the physiologies of all organs of interest simultaneously and systematically. Second, it has the ability to derive high-quality tracer input function from large arterial vessels in PET images with high accuracy for pharmacokinetic studies, avoiding invasive arterial blood sampling [9]. However, the challenge for single-bed dynamic PET imaging is that large arterial vessels are not always present in the field-of-view, and one may need to utilize other blood pools such as the carotid arteries, ascending aorta, descending aorta, or abdominal aorta [15, 16]. These approaches may involve more difficult ROI placement, and suffer from partial volume effects for smaller blood pools, such as the carotid arteries [15]. We chose the ascending aorta for obtaining the input function, as it had been determined to have the strongest correlation with the results from arterial sampling [16]. Third, the large increase in sensitivity arising from total-body coverage allows for very small amounts of activity for imaging the entire body [17, 18]. Recent study demonstrated that ultra-low activity dynamic [^18^F]FDG total-body PET scan not only obtained relevant kinetic metrics of full activity, but also reduced radiation dose and data size, making it more acceptable and easier for data reconstruction, transmission, and storage for clinical practice [11]. Therefore, half-dose ^68^Ga-DOTATATE was used in this study based on previous total-body dynamic PET data.

We found overall similar biodistribution and generally overlap of the range of ^68^Ga-DOTATATE uptake compared with previous data [19–22]. ^68^Ga-SSA distribution is limited to those tissues that actually accumulate the tracer. The high uptake of ^68^Ga-DOTATATE in the spleen, adrenals, pituitary gland, and kidneys may be associated with the high expression of SSTR2, and has been proven in previous *in vitro* studies [23, 24]. Besides, ^68^Ga-DOTATATE is excreted in the renal tract, and, therefore, renal parenchymal uptake might be overestimated due to intense excretory tracer activity in the medullary pyramids and possible signal crossover from the renal pelvis. Although *in vitro* studies have shown that hepatocytes and hepatic stellate cells of the normal liver parenchyma do not express any of the SSTR subtypes [25], high ^68^Ga-DOTATATE uptake in the liver was observed in this study. However, as an organ related to metabolism and elimination of radiotracer, nonsomatostatin receptor-mediated uptake in liver [26] may have contributed to this phenomenon.

Previous studies regarding ^68^Ga-DOTATATE biodistribution focused mainly on static imaging [21, 22], but rarely on dynamic imaging. In this study, we systematically evaluated the simultaneous biodistribution of ^68^Ga-DOTATATE over the entire body through dynamic total-body PET/CT imaging, which is the first up till now. Blood activity measurements showed that the radiopeptide was rapidly eliminated. Dynamic PET studies demonstrated that radioactivity in the blood decreased rapidly to 2.1% of the peak level within 60 min of the dynamic scan. Besides, the rapid tracer accumulation in the kidneys, followed by a passage into the bladder, indicated a main clearance way of the tracer through kidney. The ^68^Ga-DOTATATE uptake of spleen and liver increased with time, while the uptake of kidney reached the peak at 6 min followed by gradual decrease and then slow increase, which were similar to that of ^68^Ga-DOTATATE and ^68^Ga-DOTATOC in previous studies [4, 20], reflecting the combination of specific receptor binding and nonspecific tissue handling of the peptide. Unlike the protocol of 45 min dynamic scans followed by three whole-body PET/CT scans at 1, 2, and 3 hr in the literature [4, 20], 60 min dynamic protocol without longer times was used in this study. Most ^68^Ga-DOTATATE TACs of normal organs in this study were ascending, while [^18^F]FDG TACs of normal organs were descending [9]. There were essential differences in the imaging principles between ^68^Ga-DOTATATE and [^18^F]FDG, which could also be reflected by TAC characteristics.

Physiological uptake in the pancreas head has been described in ^68^Ga-SSA PET/CT imaging previously [21, 27, 28], which was also observed in this study. As shown in Figure 4, the radioactivity concentration of pancreas head was significantly higher than that of pancreas body on the basis of each time point of dynamic PET. A possible explanation is that the pancreas head is rich in pancreatic polypeptide cells, which express SSTR subtypes 1–4 on their surface [29]. This phenomenon makes differentiation between physiological and pathological ^68^Ga-SSA uptake in pancreas head challenge [21, 27]. Moreover, quantification using SUV and pancreas/liver ratio had no additional value to aid diagnosis. Whole-body dynamic ^68^Ga-DOTATOC PET/CT protocol was used to differentiate physiological uptake of the pancreatic uncinate process from pathological uptake, showing the excellent diagnostic performance of the *K*_*i*_ (90.9%) [30]. Dynamic PET scan can acquire the kinetic parameters, and might aid in differential diagnosis.

Studies on the kinetic parameters of ^68^Ga-SSA mostly focus on tumors, but rarely on normal organs. Henze et al. [5] evaluated ^68^Ga-DOTATOC kinetics in patients with meningiomas, in which the nasal mucosa was selected as the reference tissue given that it had mild to moderate physiological SSTR density expression, with the mean vB, *K*_1_, *k*_2_, and *k*_3_ values of 0.110, 0.401, 0.556, and 0.061 min^−1^, respectively. In this study, the vB (0.0009), *K*_1_ (0.057 min^−1^), and *k*_2_ (0.103 min^−1^) of nasal mucosa were much smaller, while *k*_3_ (0.077 min^−1^) was close to the above result. Because of the size of nasal mucosa, partial volume correction might account for this point.

Dynamic total-body PET imaging provides conditions for real-time and systematic visualization and quantification of various organs in the body, especially for the heart–brain axis [31]. In this study, similar kinetic characteristics among different organs were found through the hierarchical clustering analysis, which may the internal connections among these organs. However, extended study, perhaps based on related disease models, is required in the future for further explanation of the interactions and relationships of ^68^Ga-DOTATATE among different organs.

This study bears limitations. Given the standard method has not been established for clinical practice, time delay correction was not performed in this study although its importance for total-body PET kinetic modeling has been identified recently [32–34]. Second, selected patients were not healthy volunteers, but those with gNETs endoscopic resection. Therefore, discrepancy of the kinetic rates may exist between the results in this study and those from totally healthy volunteers. On the other hand, patients with gNETs endoscopic resection might have resulted in a representative referral population in current practice of patients undergoing ^68^Ga-DOTATATE PET imaging for suspected or for staging/restaging in the case of an already identified NET.

## 5. Conclusion

^68^Ga-DOTATATE uptake and clearance in different organs were different. The distribution and normal range of ^68^Ga-DOTATATE kinetic metrics in normal organs identified in this study could provide a reference for assessing tracer kinetics in future dynamic PET imaging.

## Figures and Tables

**Figure 1:** Maximum intensity projection of selected dynamic reconstructed images of a 52-year-old female.

**Figure 2:** Region of interest delineation in the (a) temporal lobe on both sides; (b) pituitary gland; (c) nasal mucosa; (d) parotid glands; (e) submandibular glands; (f) thyroid; (g) ascending aorta; (h–j) liver; (k) spleen; (k, l) pancreas; (l, m) adrenals; (n) kidneys; (o) prostate; (p) third lumbar body. RU, RM, RL, and LL in panels h to j denote the right upper area, right middle area, right lower area, and left lobe of the liver, respectively. PB and PH in panels k and l denote the pancreas body and pancreas head, respectively.

**Figure 3:** Diagram of the tracer kinetics of ^68^Ga-DOTATATE. A two-tissue compartment model is used. *K*_1_ describes the binding to the receptor, *k*_2_ the displacement from the receptor, *k*_3_ the cellular internalization, and *k*_4_ the externalization.

**Figure 4:** Time–activity curves quantified from the ^68^Ga-DOTATATE PET images of a 62-year-old male in normal organs. The injected dose of ^68^Ga-DOTATATE was 73.6 MBq. Individual symbols represent original data, and the solid line is the fit of the original data.

**Figure 5:** Three-dimensional rate constant space of three maximum likelihood clusters in normal organs. Data represent means of rate constants in each organ.

**Table 1:** Clinical characteristics of patients.

Parameters	Value
Sex	
Male	5
Female	2
Age (years)	60 (39–68)
Weight (kg)	66.2 (48.1–71.8)
BMI (kg/m^2^)	23.9 (21.1–28.4)
Gastric neuroendocrine tumor with endoscopic resection	7
Pathological grade^a^	
G1	3
G2	4
Injected dose (MBq)	69.2 (48.1–73.6)
Injected dose/weight (MBq/kg)	1.0 (0.7–1.3)

^a^According to the World Health Organization 2019 grading of gastroenteropancreatic neuroendocrine tumors. Where no units are shown, the tabulated values indicate the number of participants. Where units are shown, the values indicate the median with ranges in parentheses.

**Table 2:** Summary statistics of *K*_1_ and *k*_2_ in normal organs.

Tissues	Site	*K*_1_ (min^−1^)						*k*_2_ (min^−1^)					
		Mean ± SD	CV (%)	Intersite var. (%)	*P*	Intersubject var. (%)	*P*	Mean ± SD	CV (%)	Intersite var. (%)	*P*	Intersubject var. (%)	*P*
Nasal mucosa	Av.	0.0572 ± 0.0361	63.2	1.65	0.662	73.53	0.075	0.1025 ± 0.1209	118.0	3.86	0.501	57.45	0.282
	L	0.0507 ± 0.0255	50.3					0.2474 ± 0.5207	210.5				
	R	0.0577 ± 0.0323	56.0					0.1088 ± 0.0873	80.3				
Cerebrum	Av.	0.2102 ± 0.071	33.8	4.47	0.468	69.84	0.110	5.4444 ± 2.1166	38.9	3.81	0.503	75.95	0.056
	L	0.2058 ± 0.0639	31.0					4.4487 ± 1.8598	41.8				
	R	0.1831 ± 0.0484	26.5					3.7579 ± 1.8874	50.2				
Pituitary		0.1866 ± 0.0425	22.8	–	–	–	–	0.3077 ± 0.8121	264.0	–	–	–	–
Parotid	Av.	0.186 ± 0.1476	79.4	1.35	0.626	77.30	0.073	0.9824 ± 1.7906	182.3	1.71	0.656	65.85	0.156
	L	0.1456 ± 0.0605	41.6					0.404 ± 0.3437	85.1				
	R	0.1604 ± 0.0456	28.4					0.49 ± 0.3606	73.6				
SMG	Av.	0.2996 ± 0.1646	54.9	6.95	0.362	65.81	0.157	0.7484 ± 0.5908	78.9	0.00	0.998	47.99	0.456
	L	0.2538 ± 0.0998	39.3					0.9123 ± 0.8845	97.0				
	R	0.3287 ± 0.1838	55.9					0.9133 ± 0.727	79.6				
Thyroid	Av.	0.6024 ± 0.3092	51.3	18.85	0.121	63.64	0.186	1.5922 ± 1.0735	67.4	22.29	0.088	56.11	0.305
	L	0.6629 ± 0.2083	31.4					1.7479 ± 0.5792	33.1				
	R	0.4949 ± 0.1657	33.5					1.2023 ± 0.5193	43.2				
Liver	Av.	0.2688 ± 0.0888	33.0	26.45	0.057	17.83	0.609	0.0926 ± 0.0879	95.0	21.69	0.112	38.74	0.082
	LL	0.1775 ± 0.0844	47.5					0.0369 ± 0.0286	77.6				
	RU	0.2445 ± 0.0388	15.9					0.1235 ± 0.1154	93.5				
	RM	0.2322 ± 0.0513	22.1					0.0506 ± 0.0359	71.0				
	RL	0.2706 ± 0.061	22.5					0.0658 ± 0.0538	81.7				
Spleen		0.4864 ± 0.1385	28.5	–	–	–	–	0.0174 ± 0.0282	162.5	–	–	–	–
Pancreas	Av.	0.7439 ± 0.3157	42.4	6.21	0.390	67.35	0.138	1.9608 ± 0.951	48.5	27.30	0.055	54.38	0.336
	Head	0.5484 ± 0.4866	88.7					0.7274 ± 1.0659	146.5				
	Body	0.7409 ± 0.2997	40.5					1.8315 ± 0.8705	47.5				
Kidney	Av.	1.1767 ± 0.255	21.7	3.08	0.548	72.63	0.083	0.3823 ± 0.3048	79.7	7.17	0.355	60.22	0.237
	L	1.21 ± 0.4338	35.9					0.4786 ± 0.6549	136.8				
	R	1.0975 ± 0.2092	19.1					0.2372 ± 0.1046	44.1				
Adrenal	Av.	0.3657 ± 0.0835	22.8	5.32	0.428	33.97	0.725	0.1085 ± 0.2728	251.4	0.37	0.837	42.90	0.556
	L	0.4523 ± 0.2789	61.7					0.2766 ± 0.7318	264.6				
	R	0.3618 ± 0.085	23.5					0.2047 ± 0.5281	258.0				
Prostate		0.139 ± 0.0312	22.5	–	–	–	–	0.0594 ± 0.0696	117.1	–	–	–	–
Bone		0.1532 ± 0.0621	40.5	–	–	–	–	0.5601 ± 0.2665	47.6	–	–	–	–

SMG, submandibular gland; SD, standard deviation; CV, coefficient of variance; var., variance; Av., average; L, left; R, right; LUL, left upper lobe; LLL, left lower lobe; RUL, right upper lobe; RML, right middle lobe; RLL, right lower lobe; RU, right upper area, RM, right middle area; RL, right lower area; LL, left lobe.

**Table 3:** Summary statistics of *k*_3_ and vB in normal organs.

Organs	Site	*k*_3_ (min^−1^)						vB						Mean *R*^2^
		Mean ± SD	CV (%)	Intersite var. (%)	*P*	Intersubject var. (%)	*P*	Mean ± SD	CV (%)	Intersite var. (%)	*P*	Intersubject var. (%)	*P*	
Nasal mucosa	Av.	0.0771 ± 0.0747	96.9	10.35	0.262	42.75	0.559	0.0009 ± 0.0017	180	5.56	0.421	50.00	0.424	0.934
	L	0.7275 ± 1.427	196.1					0.0013 ± 0.0022	171.1					0.904
	R	0.0921 ± 0.0623	67.6					0.0005 ± 0.001	185.4					0.887
Cerebrum	Av.	0.0718 ± 0.0289	40.2	15.87	0.158	68.89	0.120	0.0021 ± 0.0055	264.6	7.21	0.352	45.92	0.497	0.782
	L	0.0747 ± 0.0236	31.6					0.0001 ± 0.0003	265.7					0.726
	R	0.0563 ± 0.0223	39.6					0.0034 ± 0.009	264.6					0.681
Pituitary		1.5915 ± 2.295	144.2	–	–	–	–	0.0195 ± 0.0304	155.6	–	–	–	–	0.933
Parotid	Av.	0.2817 ± 0.3589	127.4	2.01	0.629	69.19	0.117	0.0068 ± 0.0069	102.2	1.16	0.727	74.42	0.064	0.972
	L	0.1685 ± 0.1274	75.6					0.0037 ± 0.0041	111.2					0.953
	R	0.2014 ± 0.1209	60.0					0.0044 ± 0.0034	76					0.948
SMG	Av.	0.2091 ± 0.166	79.4	0.17	0.889	39.10	0.630	0.0233 ± 0.03	128.9	7.90	0.331	75.98	0.056	0.918
	L	0.2606 ± 0.3396	130.3					0.0326 ± 0.0309	94.7					0.866
	R	0.2397 ± 0.1849	77.1					0.0176 ± 0.0241	136.9					0.892
Thyroid	Av.	0.2263 ± 0.1471	65.0	7.94	0.329	72.41	0.084	0.0152 ± 0.0255	168.1	0.50	0.810	54.74	0.329	0.907
	L	0.1631 ± 0.0688	42.2					0.0176 ± 0.0153	86.9					0.833
	R	0.2204 ± 0.1322	60.0					0.0202 ± 0.0243	120					0.867
Liver	Av.	1.2921 ± 2.9613	229.2	6.71	0.637	37.47	0.097	0.0039 ± 0.0104	264.6	5.53	0.707	20.43	0.514	0.988
	LL	1.9039 ± 2.9912	157.1					0.0218 ± 0.0576	264.6					0.974
	RU	1.3334 ± 2.8644	214.8					0.0038 ± 0.01	264.5					0.974
	RM	1.2876 ± 2.9594	229.8					0.0147 ± 0.0389	264.6					0.974
	RL	0.1606 ± 0.1365	85.0					0.0027 ± 0.0072	264.6					0.972
Spleen		0.0929 ± 0.116	124.8	–	–	–	–	0.014 ± 0.024	171.6	–	–	–	–	0.988
Pancreas	Av.	0.246 ± 0.1184	48.1	4.12	0.486	54.43	0.335	0.0355 ± 0.0442	124.5	28.16	0.051	50.29	0.412	0.906
	Head	0.3371 ± 0.472	140.0					0.1627 ± 0.1669	102.6					0.834
	Body	0.206 ± 0.0999	48.5					0.0222 ± 0.0389	174.9					0.751
Kidney	Av.	0.1376 ± 0.1467	106.6	9.48	0.284	50.44	0.409	0.0076 ± 0.0099	129.9	15.63	0.161	71.94	0.089	0.930
	L	0.1424 ± 0.2001	140.5					0.0084 ± 0.0078	93.4					0.908
	R	0.0573 ± 0.0159	27.8					0.0035 ± 0.0036	102.5					0.900
Adrenal	Av.	3.3792 ± 3.0917	91.5	3.29	0.535	61.95	0.210	0.0862 ± 0.0569	66.1	27.00	0.057	54.49	0.334	0.964
	L	4.6309 ± 4.1563	89.8					0.0802 ± 0.1077	134.2					0.946
	R	3.3129 ± 3.5319	106.6					0.2489 ± 0.1824	73.3					0.896
Prostate		1.5535 ± 3.362	216.4	–	–	–	–	0.0076 ± 0.0171	223.6	–	–	–	–	0.945
Bone		0.1517 ± 0.0441	29.1	–	–	–	–	0.0089 ± 0.0077	85.8	–	–	–	–	0.807

SMG, submandibular gland; SD, standard deviation; CV, coefficient of variance; var., variance; Av., average; L, left; R, right; LUL, left upper lobe; LLL, left lower lobe; RUL, right upper lobe; RML, right middle lobe; RLL, right lower lobe; RU, right upper area, RM, right middle area; RL, right lower area; LL, left lobe.

**Table 4:** Mean rate constants of organs with similar kinetic characteristics as determined by a cluster analysis.

Group	Organs	*K*_1_ (min^−1^)	*k*_2_ (min^−1^)	*k*_3_ (min^−1^)
1	Cerebrum	0.2102	5.4444	0.0718
2	Pituitary	0.2400 ± 0.0861	0.1421 ± 0.0973	1.9541 ± 0.8308
	Liver			
	Adrenal			
	Prostate			
3	Nasal mucosa	0.4632 ± 0.3486	0.7933 ± 0.6463	0.1778 ± 0.0693
	Parotid			
	SMG			
	Thyroid			
	Spleen			
	Pancreas			
	Kidney			
	Bone			

SMG, submandibular gland. Values are presented as mean ± SD.

## Data Availability

The data that support the findings of this study are available from the corresponding author.
